# Surfactant Stock Optimization for Cost Minimization in Neonatal Intensive Care Units

**DOI:** 10.1155/2021/8346584

**Published:** 2021-12-01

**Authors:** Müfide Narli, Ali Kokangül

**Affiliations:** Industrial Engineering, Cukurova University, Adana, Turkey

## Abstract

Surfactant deficiency in newborns is a result of a respiratory insufficiency condition, which is a major cause of illness and death. In terms of maintaining vital functions that require emergency intervention, it is crucial that surfactant is available for treatment upon request. The unknown times between patient arrivals and the patients' stochastic weight changes in the hospital cause difficulties in determining the surfactant doses needed. The surfactant dose treatment for patients must be calculated according to the patient's weight. In this study, a mathematical model that minimizes the purchase, order, holding, and waste costs of the surfactant has been developed while finding the optimum vial by considering random variables such as the time between a patient's arrival and weight changes. With cost and demand affecting each other, the model uses a continuous inventory control policy, including calculating how much each preparation and vial should be used for, the reorder point, and the optimum order quantity. Also, the validity of the optimum values obtained with the mathematical model of a 66-bed neonatal intensive care unit in a hospital was tested with real data.

## 1. Introduction

An important problem for newborns, and especially premature babies, is respiratory distress syndrome (RDS). RDS is a situation of respiratory failure developing due to insufficiency of a substance called surfactant that enables the development of the lungs. RDS is seen in 40,000 to 50,000 babies in the United States alone each year [1]. In newborn intensive care units, surfactant is widely used in RDS treatment. About 115,000 surfactant doses were administered annually to neonatal RDS infants in USA [2].

Three preparations containing surfactant, beractant, calfactant, and poractant alpha are commercially available in our country. Surfactant preparations are produced from three different (origin) sources: pigs, cattle, and calves. These three different preparations of surfactant are presented in a total of five different vials. These preparations are considered to be equivalent in terms of clinical efficacy in relation to treatment. In a comparative clinical efficacy study conducted in the United States between 2005 and 2010, premature infants admitted to 322 neonatal intensive care units were treated with surfactant, and it was stated that there was no difference [3].

Treatment is applied by calculating the required amount of surfactant per the patient's weight and selecting the vial containing a sufficient amount of surfactant. Furthermore, since the surfactant in liquid form in the contents of the vials is different in milliliters in each preparation, the vials contain different amounts of surfactant material.

If one vial is not sufficient for a patient, more than one vial of the same preparation is administered. Although surfactant is the active ingredient of all preparations in clinical use, their pharmacokinetic (metabolism and excretion) properties are also different due to the different animal products from which they are obtained. For this reason, it has been stated that it is not appropriate to mix preparations with varying content concentrations [4]. In other words, when more than one vial is to be used for a patient, vials of the same preparation should be used for that patient. Following applying the surfactant drug to the patient, the surplus surfactant in the vials is recommended to be discarded without waiting [5]. Since the surfactant must be brought to room temperature before it is used, the opened vial must not be reused, as stated in the drug usage guidelines.

The doctor will determine which preparation and which vial size will be given to the patient. RDS may not be treated appropriately if the patient is given incomplete surfactant. If there is excessive administration of surfactant, it may cause serious consequences, such as not spreading to the lungs due to the volume exceeding the lung capacity and obstructing the respiratory tract as a result of overflow [6]. Due to this reason, the dose to be given to the patient must be within the tolerance range determined by calculating the patient's weight.

Surfactant application should be realized as soon as possible for babies who need it. For this reason, the medicines needed to maintain vital functions requiring urgent intervention must be accessible when requested, especially in hospitals. The specialist physician applying the surfactant treatment prefers one of the vials suitable for the patient's weight to be currently available in stock. Sometimes when the most suitable vial is not available in the stock, they have to use any available vials.

Stock management aims to maintain the stock level of drugs to meet demand and avoid stockouts. The depletion of drug stocks delays patient treatment and may have fatal consequences [7]. It is important to have the right amount of surfactant stock supplies in newborn units to make them in a timely manner to prevent these negative consequences.

The market price of surfactant drugs differs, and annual hospital treatment costs are quite high. As seen in the surfactant studies, determining the most appropriate preparation and vial size for the patient is an important issue in terms of both treatment and cost. The random changes in the time between patient arrival and patient weight over time make this problem difficult.

This problem concerns both the doctor and the hospital management. The physician tries to select the appropriate preparation and vial size. In contrast, the hospital management tries to find the proper vial size, order quantity, and appropriate order time to minimize the total surfactant cost.

When studies concerning surfactants are investigated, the studies in which surfactants are examined with respect to clinical perspective and effective cost attract attention. During the studies evaluating surfactants from a clinical perspective, Speer et al. [8] and Ramanathan et al. [9] compared poractant and beractant on RDS treatments, and the poractant performance was determined to be better clinically. Salinas-Escudero et al. [10] evaluated the treatments with surfactant and without surfactant from the cost point of view, and the results show that the treatment with surfactant is better either clinically or in terms of cost. Singh et al. [11] assessed mortality and oxygen necessity during the evaluation of clinical effectiveness of surfactants in RDS treatments.

Similar studies have compared the cost per patient of double or triple beractant, calfactant, and poractant alpha combinations. However, these studies do not have methods for reducing the cost of work or making improvements. Surfactant treatments on patients are evaluated by cost per patient, factors that affect costs, and benchmark results. Marsh et al. [1]; Brown et al. [12], Zayek et al. [13]; and Sekar et al. [14] obtained different results in their assessments for the effective cost. Some studies focused on beractant and poractant. Brown et al. [12] concluded that beractant was more appropriate from a cost-effective perspective, and for Marsh et al. [1], poractant was more appropriate. When Zayek et al. [13] evaluated calfactant and poractant in their study, they concluded that calfactant is cost-efficient. Sekar et al. [14] concluded that the cost-effectiveness analysis of calfactant, poractant, and beractant is close, but beractant has a lower cost.

Brown et al. [12] and Sekar et al. [14] both assessed clinical benefits and cost-effectiveness. Brown et al. [12] put forward that clinical evaluations of poractant and beractant show that poractant is more efficient in terms of the duration of hospital stay and respiratory support. Sekar et al. [14] studied the clinical superiority of calfactant, poractant, and beractant and concluded that calfactant has a lower mortality rate. Poractant and beractant have equal mortality rates, but in ventilation, poractant has superiority.

Marsh et al. [1] studied cost-reduction analysis and compared the cost-effective profiles for beractant and poractant. The analyses used with the three models were based on single- or multiuse vial scenarios, average wholesale costs, and calculation of price per patient. Model one contained a single-dose vial and the average weight of the babies. Models two and three were developed based on clinical data from two previously published studies from Speer et al. [8] and Ramanathan et al. [9].

Brown et al. [12], Zayek et al. [13], and Sekar et al. [14] calculated the average drug cost per patient case for the treatment of neonatal RDS in their surfactant-related cost-effectiveness studies. Clinical results were statistically compared for the duration of respiratory support treatment, the duration of hospital stay, and the development of complications with these drugs.

In the literature search related to surfactants, studies on surfactant stock management were not found. For this reason, studies on stock management were examined in general. This study recognized that stock management problems are classified according to many factors, such as deterministic or stochastic stock parameters, continuous review and periodic review stock control, and single-piece multipart stock.

Classification of stock models as deterministic and stochastic depends on whether certain variables are random or not. These variables are usually constituted of demand and lead time. In deterministic models, these variables are considered constants, and stock depletion is not allowed if necessary. Zheng [15] stated that when the demands for the stock system are evaluated as stochastic processes, it generally gives more accurate results than the deterministic EOQ model. It has been stated that deterministic models, in which the demand is certain, are far from the problems encountered in real life. Therefore, stochastic models, in which the variables are random, are more commonly used. In our study, the random variation between patient visits and patients' weights over time necessitates the stochastic modeling approach in surfactant stock optimization.

Stochastic models are classified as periodic or continuous reviews as per the inventory control frequency. As surfactant is perishable and costly, using a continuous control approach in stock optimization is more suitable. Therefore, the stock policy of continuous review was taken into account in our study.

There are certain studies in the literature in which continuous control policies are implemented. Azimi et al. [16]; Axsäter [17]; Moinzadeh and Nahmias [18]; and Federgruen and Zheng [19] used the continuous review inventory policy (*Q*, *r*) approach in the studies they conducted. As stated in Federgruen and Zheng's [19] study, according to the policy of continuous stock control (*r*, *Q*), the policies where stock is constantly reviewed and a fixed quantity of *Q* is ordered as soon as the stock level drops at the reorder point, *r* is the most suitable policy for one-piece stock systems. In their inventory modeling study, in which he also considered the storage cost, Moinzadeh and Nahmias [18] made a one-piece continuous review inventory model when demand is stochastic, and there is storage space constraint. In Axsäter's [17] stochastic demand and single-stage inventory model, delivery time and demand are taken as normal distribution. It aimed to minimize the holding and ordering costs by considering those costs and occupancy rate constraints.

In the literature review, studies on drug stock management were searched, and few studies were found. Li et al. [20] stated that drug stocks have a short shelf life due to their perishability, and, therefore, drug stocks should be managed effectively. However, it has been emphasized that many uncontrollable factors can lead to random delivery times of drugs. In this study, a stock model was created that takes into account the deterioration of drugs and stochastic delivery time, and the demand is assumed to be constant. Pharmaceutical inventory management has developed a mathematical model to increase the turnover rate of drugs, reduce inventory costs, and prevent errors. In his study, Saha and Ray [21] stated that current stock models for drugs in the health field generally accept demand as a random variable independent of environmental factors. However, it was thought that various randomly changing factors could have a significant impact on the demand for drugs, such as the changing condition of the patient, the patient's ambiguous response to treatment, the uncertain length of the hospital stay, and the transition from one type of hospital care unit to another at different treatment stages. In the study, the Markov decision process model provided the inventory cost minimization, taking into account the (s, S) stock control policy, and the results were evaluated.

It attracts interest that cost-based inventory models in the literature are stochastic rather than deterministic. But stock policies are followed in all models, and the differences in applications create differences for each problem. In the modeling process, it is vital to consider all the features of the problem and model them in accordance with real life.

In this study, stochastic stock modeling was developed by considering continuous control policy and demand uncertainty. Demand uncertainty is correlated with patient arrivals and patient weights and is also affected by drug prices. The particular way that the demand in the study is formed makes our study different from other studies in the literature. In the model we created, the waste cost was minimized along with the stock costs, and it was determined that a drug use policy was formed according to the results obtained. In addition, the drug use policy, which is formed according to the results obtained, is presented.

The annual treatment costs of surfactant drugs in the hospital are changing, and the market prices of the units are quite high. Major problems emerge regarding both treatment and cost for the most appropriate preparation for each patient and determining the vial size, as seen in surfactant-related studies. The time between patient arrivals and the random changes in patients' weights over time complicate this problem. This problem can be solved with a mathematical approach that considers the stochastic changes and the interactions between demand and cost.

This problem concerns both doctors and hospital management. Doctors decide which preparation and vial size should be given to each incoming patient, and hospital management tries to decide how much of each preparation and vial size to order. Both cases look to minimize the total cost of surfactant, which is a difficult problem to solve.

In this study, a mathematical model has been constructed to find economical order sizes and the optimum vial type to be given to each patient and minimize the cost of the surfactant according to determined restrictions. Steps followed up in the study are given below:

  Determining the limitations related to surfactant treatment applications.
  Examining the stock policy applied in the intensive care unit of the hospital where the study was conducted.
  Gathering inventory cost information.
  Obtaining and organizing patient arrival and weight data from the hospital to determine the drug demand and finding appropriate probability distributions.
  Establishing the constrained mathematical model.
  Solving the mathematical model, whose purpose and constraints are determined, in a suitable computer package program and evaluating the results.
  Establishing the simulation model to test the mathematical modeling approach with the simulation approach.
  Testing the validation and verification of the simulation model.
  Comparing the mathematical model with the simulation model results for testing.

## 2. Mathematical Modeling Approach

Surfactant treatment is applied with dose calculations as mg/kg, depending on the patient's weight. However, the amount of surfactant in each preparation, the vial sizes, and the costs are different.

The preparate and vial size to be applied to the patient depends on the doctor's decision. If the doctor cannot find the appropriate preparations of vials in stock, based on the patient's weight, then the doctor may have to use any of the current vials. Therefore, deficiency in planning stocks affects both treatment and costs. This creates a major problem for deciding which preparations and sizes should be purchased, how many should be purchased, and when they should be purchased.

It is possible to model this problem as an inventory optimization problem. Therefore, the first step should be deciding how to apply a stock policy. Accordingly, since the material is medicine and there is a deterioration feature of the drugs, a continuous stock control policy can be applied. According to this policy, an order should be placed with the optimum order amount when the stock falls to the reordering level for each vial, and the stock level for each surfactant preparation should be controlled continuously.

The structure of the problem is seen as a classic inventory problem, but it also includes the costs of inventory and drug waste. Also, because of the randomness of the arrival times of patients who need surfactant and the randomness of incoming patients' weights, the drug needs according to weight occur randomly. This problem shifts away from a classic economic inventory model (EOQ) and comes closer to a restrictive nonlinear mathematical modeling approach. The proposed notations and decision variables used in the mathematical model are given below.

### 2.1. Notation

 
*t*:1, 2, ..., *m*—time index (day)
 
*i*: 1, 2,…, *n*—patient index
 
*j*: 1, 2, ..., *s*—preparation index
 
*k*: 1, 2, ..., l—vial size index
 
*C*_*jk*_: the unit price for the vial *k* of preparation *j* ($/per)
 
*FS*_*jk*_:*j*—the amount of surfactant in the vial *k* of preparation *j* (mg/vial)
 
*OC*_*jk*_: ordering cost for vial *k* of preparation *j* ($)
 
*h*_*jk*_: holding cost for the vial *k* of preparation *j* ($/unit-year)
 
*BW*_*ti*_: patient *i* of birth weight at day *t* (kg)
  TA: time of arrival between patients (day)
 
*n*_*jk*_: number of orders of preparation *j* and vial *k* annually
  MD: minimum dose ratio (%)
  KS: the amount of surfactant to be given to the patient per kg unit (mg/kg)
  M: a large positive number
 
*Y*_*tij*_: at day *t*, the status of preparation *j* using or not using for patient *i*
 
*SR*_*ti*_: at day *t*, need of surfactant for patient *i*
 
*D*_tjk_:at day *t*, demand of preparation *j* and vial *k*
 
*DT*_*jk*_:the total annual demand for vial *k* of preparation *j*
 
*W*_tijk_: at day *t*, for patient *i*, waste drug amount of vial *k* of preparation *j* (mg)
 
*CW*_*jk*_: cost waste for vial *k* of preparation *j* ($/mg)
 
*P*_*ti*_: waste drug amount of patient *i* at day *t*
 
${\hat{d}}_{jk}$: the maximum daily demand for vial *k* of preparation *j* (mg/day)
 
${\hat{L}}_{jk}$: the maximum acquisition time for vial *k* of preparation *j* (day)

### 2.2. Decision Variables

 
*X*_tijk_:at day *t*, given to patient *i*, preparation *j* and *k*, using the number of the vial (unit)
 
*Q*_*jk*_: the ordering amount for vial *k* of preparation *j* (unit)
 
*R*_*jk*_: reorder point for vial *k* of preparation *j* (unit)

The main purpose of this study is to find the optimal order quantity of surfactant (*Q*_*jk*_) to obtain the minimum cost for the total surfactant usage. Considering the structure of the problem, it looks like a classical economic order quantity model. However, in an application, it should optimize EOQ and optimize for each patient, the type of drug, which size, and how many vials should be given. To reflect this expectation of the model, the following assumptions, which are effective in surfactant applications, should be taken into account.

### 2.3. Assumptions

In the construction of the mathematical model, the following assumptions were taken into consideration.

  The same patient may require the implementation of more than one surfactant. In this study, surfactant treatments applied to the same patient are taken independently of each other.
  If one vial is not sufficient for surfactant treatment regarding the same patient, treatment can be completed with another vial for the same preparate.
  Each preparations' clinical effectiveness is equal.
  Leftover drugs from a combo box cannot be used for another patient; leftover drugs are thrown out.
  The medication dosage to be given to each patient is calculated by the unit weight of the patient.
  It is required to give each patient at least a certain percentage (MD) of surfactant need.
  The purchase price does not change during the planning period.
  It is accepted that orders were delivered at the same time.
  Cut of stock is not allowed.
  Holding cost does not change over time.

Under these assumptions, the optimal order quantity (*Q*_*jk*_, ∀*j*, *k*) will be found, which minimizes the total cost of surfactant (TC) used in the NICU.

### 2.4. Objective Function

(1) $$\begin{array}{c} \text{Minimize }TC=\sum_{t}^{m}\sum_{j}^{s}\sum_{k}^{l}C_{jk}D_{tjk}+\sum_{t}^{m}\sum_{j}^{s}OC_{jk}\left(\frac{DT_{jk}}{Q_{jk}}\right)+\sum_{j}^{s}\sum_{k}^{l}h_{jk}\left(\frac{Q_{jk}}{2}\right)+\sum_{t}^{m}\sum_{i}^{n}\sum_{j}^{s}\sum_{k}^{l}W_{tijk}CW_{jk}\text{. } \end{array}$$

Constraints:

(2) $$\begin{array}{c} SR_{ti}=KS\left(BW_{ti}\right);\;\forall t,i, \end{array}$$

(3) $$\begin{array}{c} \sum_{j=1}^{s}\sum_{k=1}^{l}X_{tijk}\left(FS_{jk}\right)\geq M\;D\left(SR_{ti}\right);\;\forall ,t,i, \end{array}$$

(4) $$\begin{array}{c} Q_{jk}\leq \sum_{t=1}^{m}D_{tjk};\;\forall ,j,k, \end{array}$$

(5) $$\begin{array}{c} \sum_{i=1}^{n}X_{\text{tijk}}=D_{\text{tjk}};\;\forall ,t,j,k, \end{array}$$

(6) $$\begin{array}{c} DT_{jk}=\sum_{t=1}^{m}D_{\text{tjk}};\;\forall ,j,k, \end{array}$$

(7) $$\begin{array}{c} \sum_{j=1}^{s}\sum_{k=1}^{l}\left(X_{\text{tijk}}\right)\left(FS_{jk}\right)-SR_{ti}=P_{ti};\;\forall ,t,i, \end{array}$$

(8) $$\begin{array}{c} \text{Eer}\overset{⌣}{g}P_{ti}\leq 0\text{ ise}W_{ti}=0;\;\forall t,i, \end{array}$$

(9) $$\begin{array}{c} \text{Eer}\overset{⌣}{g}P_{ti}>0\text{ ise}W_{ti}=P_{ti};\;\forall t,i, \end{array}$$

(10) $$\begin{array}{c} n_{jk}=\frac{DT_{jk}}{Q_{jk}};\;\forall ,j,k, \end{array}$$

(11) $$\begin{array}{c} R_{jk}=\left({\hat{d}}_{jk}\right){\hat{L}}_{jk};\;\forall ,j,k, \end{array}$$

(12) $$\begin{array}{c} X_{\text{tijk}}\geq 0\text{ integer},\;\forall ,t,i,j, \end{array}$$

(13) $$\begin{array}{c} W_{\text{tijk}}\geq 0;\;\forall ,t,i,j,k, \end{array}$$

(14) $$\begin{array}{c} Y_{tij}=\left\{\begin{array}{c} 1\text{ If, at day }t\text{, patient }i\text{ has }j\text{ kind of preparation,}\\ \text{0 If, at day }t\text{, patient }i\text{ has not }j\text{ kind of preparation,} \end{array}\right) \end{array}$$

(15) $$\begin{array}{c} \sum_{j}^{s}Y_{\text{tij}}\leq 1;\;\forall t,i, \end{array}$$

(16) $$\begin{array}{c} \sum_{k=1}^{l}X_{\text{tijk}}\leq Y_{\text{tij}}\left(M\right),\;\forall t,i,j. \end{array}$$

In the study, as seen in the objective function of equation (1), annual surfactant stock cost is considered; the four cost types are purchase, order, holding, and drug waste. The coefficients used in the objective function are explained as follows. Purchasing cost (*C*_*jk*_) is the market price, and in this model, it changes based on preparation and vial types. Ordering cost (*OC*_*jk*_) is the cost of preparing and expenses from the purchasing stage until delivery. The ordering cost is independent of the order quantity, and it is constant [22]. Holding cost (*h*_*jk*_)  for stock includes storage, protection, obsoletion, insurance, maintenance, and depreciation, including the interest that connects to such, as the cost of inventories may include other costs. Holding cost is calculated according to the unit price of the inventory item; it is usually considered to be 15–20% of the unit price [22].

For each patient, opened vials sometimes contain a larger dose than the patient needs. After the surfactant application, the remaining medication in the vial must be discarded immediately and cannot be used on another patient. This leads to drug waste and increased costs and affects the preparation and vial size selection. Therefore, the objective function (1) considers the cost of waste as a factor.

The amount of the surfactant (*SR*_*ti*_) to be applied to each patient according to the patient's weight is calculated as seen in equation (2). Each patient's surfactant need is calculated according to the patient's weight, but in practice, the calculated dose can be applied in a specific proportion (*MD*) as a missing dosage. This situation is shown in equation (3). Not all manufacturers produce the same vial size *(k)* and content (*FS*_*jk*_), which is expressed in equation (3). The ordering amount (*Q*_*jk*_) can be a maximum annual demand for each preparation and vial size. This situation is shown in equation (4). The constraint for meeting the daily demand of each preparation and vial is shown in equation (5), and the total annual demand amount is shown in equation (6).

Each vial contains *FS*_*jk*_ and surfactant amount *SR*_*ti*_, whereas (2) shows patients' needs and the differences between them as a positive number shown as *P*_*ti*_ in equation (7). The value of *W*_tijk_ can be negative because the surfactant needs of the patient (*SR*_*ti*_) are less, as the MD value in equation (3), and the maximum MD value is less, as an application of surfactant. Since the values of *P*_*ti*_ that can take positive and negative values are only constituted of positive values, values greater than zero are taken as *W*_tijk_, whereas for *W*_tijk_ to take positive values, a relevant situation is provided in equations (8), (9), and (13).

*W*_tijk_ is calculated as the amount of waste in mg. The cost of the surfactant amount (mg) in each preparation and vial cost are found with *C*_*jk*_/*FS*_*jk*_. As seen in equation (1), the waste cost that will occur throughout the year is found with the multiplication of waste amount formed with waste cost *C*_*jk*_/*FS*_*jk*_.

The annual number of orders is given in *n*_*jk*_ (equation (10)). In this study, assuming that stocks will not be allowed to be cut, the reorder quantity (*R*_*jk*_) is expressed in equation (11). *R*_*jk*_ value is calculated for the reordering amount in the ${\hat{d}}_{jk}\;$ case where the maximum possible lead time $\left({\hat{L}}_{jk}\right)$ and daily surfactant demand is the highest. The number of each vial given to a patient is shown as an integer state in equation (12). The preparation's ability to be or not be given to a patient is shown as a binary variable in equation (14).

The obligation for a complement treatment preferring the same vial preparation is shown in constraint equations (15) and (16). This happens when a vial is opened and does not meet the required surfactant treatment dose for a patient's weight. *M* is a large positive number used to remove the possibility of going to the infinity of *X*, which is an integer variable.

The lead time $\left({\hat{L}}_{jk}\right)$ is the time between order placement and delivery. Lead time can be fixed or stochastic. In the study, the lead time varies between the same day or three days.

In this study, reordering amount (*R*_*jk*_) is shown in equation (11) because it is assumed that the stock cut will not be allowed. The possibility of the supply period is the highest $\left({\hat{L}}_{jk}\right)$ time, and when the daily demand for surfactant is the highest $\left({\hat{d}}_{jk}\right)$, there are the reordering amount and annual ordering number (*n*_*jk*_) in equation (10).

It is not enough to minimize stock cost only for finding which patient should take which preparation or how many vials are in this independent stock policy study. For this reason, in addition to the purchase price of the drug, the ordering, holding, and cost of drug waste were taken into account.

In this constructed mathematical model, the purpose is to find the minimum total cost value (equation (1)) under the same constraints (equations (2)–(16)). As a result of the solution, the model for each patient can account for which preparation and vial size (*X*_tijk_) will be obtained. Also, the reorder level (*R*_*jk*_) for each vial and type of preparation as well as the total (purchase, order, holding, and waste) cost can be found as the minimum cost with ordering size (*Q*_*jk*_).

Hospital management should constantly observe each preparate and vial size in the store, and if the drug stock level decreases to the optimum reorder point (*R*_*jk*_ ), then they should order as much as the obtained optimum order amount (*Q*_*jk*_). Thus, the total surfactant cost should be minimal.

Even though the probability distributions of the time between patient arrivals from hospital records in past years and the patient's weight are taken into account in the construction of the mathematical model, the patient arrivals and weights that will occur in the year of application may not be the same. This may cause a slight deviation in the application of (*R*_*jk*_) and (*Q*_*jk*_) of the results we obtained with the mathematical model. For this reason, it should be determined whether the results obtained in the study are compatible with real life and how they will be applied in practice.

Results for the validity check of the mathematical model and the application for the real-life planning period can be obtained, and the results can be compared with the model results. However, this will be possible after a long period—at least one year—of model results. Another way to test the model is by implementing the simulation approach.

## 3. Simulation Model

The total cost of surfactant *(TC)* can also be obtained by a simulation model with the optimal values of *X*_ijk_, *Q*_*jk*_, and *R*_*jk*_, which are obtained from the mathematical model that considers the same model assumptions, the time between patients' arrivals, and the probability distributions of patient weights.

In the constructed simulation model, surfactant can be applied to each patient according to the size of the preparation and vial that should be given according to the patient weight class from the mathematical model. If the amount of the surfactant preparations in stock for each of the vials—which is controlled continuously—decreases to the *R*_*jk*_ value, then it will order the *Q*_*jk*_ amount.

The solution of the simulation model can be found in software packages such as ARENA software. The length of the simulation is the time for the simulation model to calculate the performance criterion. There is a tradeoff between the number of replications and the simulation length. Therefore, the adequacy of the number of replications of the study should be tested.

In determining the number of replications in the analysis of the simulation output by using the relative error (*γ*) formula, the adequacy of the number of replications should be tested. The relative error and the number of replications can be calculated with equation (17), and the relative error can be calculated by the corrected relative error formula in equation (18) [23].

(17) $$\begin{array}{c} n_{r}^{*}\left(\gamma \right)=\min\left\{i\geq n:\frac{t_{i-1,1-\propto /2/\sqrt{s\left(n\right)/i}}}{\left|\bar{X}\left(n\right)\right|}\leq \gamma^{\prime }\right\}, \end{array}$$

(18) $$\begin{array}{c} \gamma^{\prime }=\frac{\gamma }{\left(1+\gamma \right)}. \end{array}$$

For sufficient replication to determine the count, at least ten replications should be performed initially. For better solutions, it is preferred for the cardinality (∝) value and the relative error (*γ*) to have a value of 1–5% [24].

If the mathematical model and simulation approach results are compared according to the percentage of the value of compliance, the validation of the mathematical model can be tested. If the value of compliance is found to be high, then it will show that the two approaches give similar results and validate the tested model.

## 4. Case Study

The retrospective application of this study took place in an important part of a large hospital; the hospital has a capacity of 143 beds, 66 of which are for the NICU. The data retrieved from the hospital database was used with the permission of hospital management. The data accounted for 3,086 patients in the NICU for approximately 24 months between September 11, 2016, and October 28, 2018. Surfactant applications occurred 413 times with these patients. During hospitalization, there was a need for repeated surfactant treatment in patients.

The data used in the hospital is from three different preparations (*j* = 3) offered on a commercial basis in five vial sizes (*k* = 5), as shown in Table 1. Every preparation unit, in ml, has a different amount of surfactant preparation inside. Also, each preparate offers different vial sizes. For example, beractant is only produced in 8 ml per vial. This vial contains 200 mg of surfactant and, therefore, contains 25 mg/ml of surfactant. The application of surfactant is given according to the incoming patient's weight in the hospital; for one kg of weight, they are given surfactant with *SR*_*ti*_= 100 mg. As seen in Table 1, poractant and calfactant have two vial sizes. The details about these vials are given in Table 1. As seen in Table 1, constraints (19, 20, 21) must be added in each preparation to reflect this situation in the model.

(19) $$\begin{array}{c} X_{\text{tijk}}=0;\;\forall ,t,i;\;j=1;\;k=2,3,4,5, \end{array}$$

(20) $$\begin{array}{c} X_{\text{tijk}}=0;\;\forall ,t,i;\;j=2;\;k=1,4,5, \end{array}$$

(21) $$\begin{array}{c} X_{\text{tijk}}=0;\;\forall ,t,i;\;j=3;\;k=1,2,3. \end{array}$$

The probability distributions of both the time between patient arrivals and patient weights were analyzed with the Kolmogorov–Smirnov test. As a result, the incoming patients did not fit into any theoretical statistical distribution. For this reason, an experimental distribution was applied to patients' arrivals. It was determined that the observed daily patient visits ranged from 0 to 9 patients. Therefore, the interval value (*n*) is taken as *n* = 10 since there are ten different observations. By considering the number of patients coming every day in the study, the number of patients per day was taken as a class. In this respect, the class determination was made easily. After the interval values were determined, the number of observations (frequency) was calculated.

Incoming patient weights were found to fit a lognormal distribution according to the Kolmogorov–Smirnov test, with a *P*-value = 0.129 and 0.18 + LOGN (1.71, 1.31). This result obtained is shown in Figure 1.

The time between consecutive patient arrivals and the probability distribution of daily weights (*t*), the number of patients who will arrive at the hospital (TA), and these patient's weights (*BW*_*ti*_) are obtained. *BW*_*ti*_ is the weight distribution for patient *i* at day *t*, and the amount of surfactant required according to this weight distribution will be obtained with the *SR*_*ti*_ in equation (2). Surfactant treatment for every patient in the hospital has a dose of 100 mg/kg. The hospital normally obtains surfactant needs (*SR*_*ti*_) according to a patient's weight; however, they can allow lower amounts than that for patients. The hospital taken into consideration gives patients at least 75% of a needed drug. Therefore, in equation (3), the MD value is taken as 75%. The hospital management wants to take stock planning for one year, so *t* is equal to 365.

As a result of considering the constructed theoretical model, the application is made for the hospital's mathematical model. The resulting application model is obtained as shown in Table 2 by using GAMS package software. The optimum results are found in 2.09 seconds with a computer with Core i7 3.66 MHz and 326 RAM.

The amounts of each type of surfactant and the vial sizes in the store are constantly checked. When the stock level reaches the reorder point (*R*_*jk*_), in Table 3, the order should be placed for the value of *Q*_*jk*_, which is obtained from the optimum order amount for the hospital. In this case, the annual surfactant cost will be minimized (TC = $21,720.99).

The results for each patient that came within the year with constraints 2–19 and with optimum administration of medication are shown in Table 3. For beractant (*DT*_11_), there is no need; poractant's second vial (*DT*_22_) shows an amount used of 148; for *DT*_23_, there is no need; calfactant's fourth vial (*DT*_34_)shows an amount used of eight, and for the fifth vial (*DT*_35_), the amount used was 31.

Another result of using the mathematical model under variables 2–18 during the planning period is that the total cost (TC) of what needs to be given to each patient should be minimized by selecting an appropriate preparation and vial size. According to this result, the planning period determined that 128 patients have surfactant applications annually. Patients who were treated with surfactant therapy in the first month have the mathematical model results shown in Table 2. For example, according to the mathematical model, a surfactant application in *t* = 4 when the patient weight is 1.539 kg means the patient should take the second flacon, which is the result of the minimum cost model.

The results of the mathematical model, daily patient arrivals, vial applications, and preparations obtained are shown in Table 2. These results were edited according to Table 2, which shows that vials are assigned to patients according to weight class. As seen above, for any of the vials that should be given for any weight, the appropriate vial can be found. For example, for an infant of 3.023 kg who came in at day 30, which vial should be given to the infant can be found. In the table, according to the weight of the infant included in the sixth class—since *n* is the number of poractant preparations—it is shown that vial two should be given.

As per the mathematical model results, below Figure 1 is obtained when the graphical distribution of the patient weight and the preparation used is examined. As seen in the model results, which minimizes the waste and stock costs, certain vials are used intensively in certain weight ranges. This situation is seen in Figure 2.

As shown in Figure 2, it is possible to state that certain vial assignments are made at certain weights. When the model results are assessed, the vial assignments made according to weight are classified as shown in Table 4 below.

Considering the one-year study period of the model, the optimal preparation and vial sizes that should be applied to each patient within this period are taken into account, and the surfactant used depending on the patient's weight is divided into six classes, and Table 4 is arranged. In the model application, the patient's weight class should be found, and then the preparation and vial on the table should be applied.

According to the mathematical model results, the total surfactant cost will be minimized in the future and in real life when the most appropriate vial is applied for each patient using the patient weights in Table 4. The optimum drug use is given in Table 4, with the probability distributions of the time between patients' arrivals and patients' weights, to test the applicability of the mathematical model results to the hospital. The simulation model is constructed based on the control stock policy, according to *Q*_*jk*_ and *R*_*jk*_ values. The proposed simulation model is given in Figure 3.

The length of the simulation proposed in the mathematical model was selected as 365 days. By conducting a replication compliance test, which runs 30 replications in the simulation model ARENA, results are found and shown in Table 2. First, ∝ = 0.05 and *γ* = 0.05, and according to equation (18), *γ*′=0.047, and equation (15) shows *n*_*r*_^*∗*^(*γ*)=0.04. As a result, 30 replications are enough because *n*_*r*_^*∗*^(*γ*) ≤ .

## 5. Comparison of Mathematical Model and Simulation Model Results

In the study, to compare the simulation results with the mathematical model results, conformity percentage values of the mathematical model results and simulation model results were calculated. The conformity percentage results of the mathematical model and simulation approach can be seen in Table 5. These results are obtained by using the following equations:

(22) $$\begin{array}{c} \text{Absolute Eror}=\left|148-156\right|, \end{array}$$

(23) $$\begin{array}{c} \text{Relative Error}=\frac{\left|8\right|}{148}, \end{array}$$

(24) $$\begin{array}{c} \text{Percentege Error}=\text{Relative Error}*100, \end{array}$$

(25) $$\begin{array}{c} \text{Conformity Percentage}=\left(100-\text{Percentage Error}\right)=94.59. \end{array}$$

As shown in the first line of Table 5, the mathematical model gives an optimum value of 148 poractant; however, the simulation model shows 156. According to these results, the agreement rate of the mathematical model and simulation model poractant demand results was 94%, as given below.

In Table 5, conformity is at 50% for analyzing the results of the request for annual surfactant; the compliance rate for the fourth calfactant vial decreased by 50%. However, the preparation of aggregate demand (*DT*_*jk*_) was 187; that share is low, at 8/187. Therefore, the compliance percentage is low for poractant; this drug has a low application percentage, so it also has a low effect. The conformity is 91.98% in Table 5. This shows quite a good conformity considering the total annual demands.

As a result, Table 5 has more than 90% conformity for the total preparation and vial numbers, the number of incoming patients, and total cost results. In this study, the presented approach based on mathematical modeling in real life has 90% conformity.

## 6. Results

In the mathematical model, the amount of medication that should be provided to each patient was integrated with the optimum order for the first time. In the model, purchasing, stock, order costs, and waste drug costs were taken into account simultaneously.

In the study, grouping the patient weights obtained from the model and determining the vial to be given to each weight group will enable the model to be used easily in practice. The only thing necessary in the application is to look at the weight class, including the weight of each patient randomly, and apply the optimum preparation and vial size suggested by the model for that weight class.

These results will provide a great convenience for the physician applying the surfactant treatment in terms of vial selection. Hence, during the surfactant application, the model's applicability will be practical. The doctor can choose according to these intervals without thinking about which vial will minimize the cost at the bedside. In the mathematical model that is constructed, the amount of surfactant given per unit kilogram, the dose rate at which the surfactant can be incompletely used, drug purchasing, and costs are entered as a parameter.

Another important result of the study is stock optimization. For this purpose, all that the hospital management needs to do is to observe the drug stock level for each preparation and vial size, and when the stock level drops to the ordering point, the order can be placed according to the optimum order quantity (*Q*_*jk*_) suggested by the model. Hence, stock and waste costs will be minimized at the same time.

This study found the optimum preparation type and vial size, which should be given to minimize the total drug cost, according to the objectives and constraints determined by considering the continuous stock control policy.

In this study, a single-item, continuous review (*R*, *Q*) stock control model was developed as a stock model, including stochastic demand. Demand varies according to the cost of the drug used depending on the patient and weight. Stochastic demand changes depending on the cost. This is the most distinguishing feature of this study compared to other studies.

With this model, cost-effectiveness will be achieved in practice in terms of stock costs and decisions in stock management. With the determination of optimum surfactant stock orders, overordering and underordering costs will be prevented. Holding costs due to excess stock will increase stock costs, and insufficient stock may cause a pause in the treatment process. As a result, it may cause irreparable consequences or even death due to the inability to intervene in the intensive care patient on time. With this model, the realization of this situation and costs can be prevented.

Regarding solution results of this mathematical model, which aims at cost minimization, different results can be obtained by changing the values of the determined parameters. In this case, the only thing to do is repeat the solution by including the current parameter values in the theoretical model. Thus, different results can be obtained with different parameter values that may arise from differences in practice or treatment. There are some differences in surfactant dosing and treatment practices in the neonatal guidelines of countries.

The time in the model was annual, and annual results were obtained. The model can also be run for several years, and its results can be evaluated. In fact, the desired period can easily be changed daily, weekly, and monthly, and the results can be evaluated. Since the surfactant demand obtained in the results and the required optimum stock amounts are determined, it is thought to be very useful in stock policy, purchases, and managerial decision processes.

The validity of the constructed mathematical model was tested with the simulation model, and the results were compared. The fit value is higher than 90%, indicating that the two approaches yielded similar results and validated the tested model. When the results of the mathematical model and simulation approach were compared, it was found that the mathematical model overlapped by testing its validity according to the % fit value.

## 7. Suggestions

In this study, three different preparations were taken into consideration and presented to the hospital. In this case, the annual cost of waste increased by 7% of the surfactant cost. Optimization studies could minimize this ratio, which manufacturers could do on each preparation vial amount and size. Such a study would reduce the drug cost and thus facilitate access to the drug for some patients and, at the same time, increase the efficiency of drug use.

## Figures and Tables

**Figure 1:** Weight distribution of patients undergoing surfactant treatment.

**Figure 2:** Weight of patient and used preparation.

**Figure 3:** Simulation model.

**Table 1:** Data on surfactant drugs.

Preparation (*j*)	Type of vial (*k*)	Vial size (ml)	Surfactant dose (mg/kg)	Surfactant amount (mg/ml)	Total surfactant in the vial (mg/flacon)	Cost of one vial *C*_*jk*_ ($/flacon)	Waste cost *CW*_*jk*_ ($/mg)	Order cost(*OC*_*Jk*_) $/order	Holding cost (*h*_*jk*_), $/year-unit
Beractant	1	8	4	25	200	210,2	1,05	25	30.2
Poractant	2	1,5	1.25	80	120	87,38	0,72	25	13.05
	3	3	1.25	80	240	222.2	0.925	25	33.3
Calfactant	4	3	3	35	105	107,61	1,025	25	16.2
	5	6	3	35	210	160.95	0.76	25	24.15

**Table 2:** Daily incoming patients' weights and application of preparation and vials to patients.

Day	Incoming patients (day)	Weight of patients (kg)	Preparations				
			Beractant	Poractant		Calfactant	
			Used vials				
			1	2	3	4	5
4	1	1.539		1			
8	1	1.364		1			
9	6	2.040					1
		3.992			2		
		1.022				1	
		0.999		1			
		2.605					1
		1.234		1			
14	1	1.798					1
22	1	1.888					1
27	1	2.197					1
30	1	3.023					2

**Table 3:** The mathematical model results for each preparation and vial size.

Preparation (*j*)	Vial (*k*)	*DT*_*jk*_(unit)	${\hat{d}}_{jk}$ (unit)	${\hat{L}}_{jk}$	*Q*_*jk*_(unit)	*R*_*jk*_(unit)
Beractant (1)	1	—	—	—	—	—
Poractant (2)	2	148	9	3	24	27
	3	—	—	—	—	—
Calfactant (3)	4	9	1	3	5	3
	5	31	4	3	8	12

**Table 4:** Patient weight class ranges determined according to the results of the mathematical model.

Class	Interval of patients' weights	Used preparation and vial (per)
1	≤0.999	Poractant, second vial
2	1000–1188	Calfactant, fourth vial
3	1189–1641	Poractant, second vial
4	1642–2099	Poractant, from second vial, two units or calfactant, fifth vial
5	2100–2768	Calfactant, fifth vial
6	2769 and more	Poractant, second vial *x n* units

**Table 5:** The mathematical model and simulation approach conformity percentage results.

Preparation (*i*), vial (*j*)	Mathematical model (unit)	Simulation model (unit)	Absolute deviation	Percentage error	Conformity percentage
Beractant (*i* = 1, *j* = 1)	—	—	—	—	—
Poractant (*i* = 2, *j* = 2)	148	156	8	5,405	94, 59
Poractant (*i* = 2, *j* = 3)	—	—	—	—	—
Calfactant (*i* = 3, *j* = 4)	9	12	4	50	50
Calfactant (*i* = 3, *j* = 5)	31	34	3	9,67	90, 33
Total number of patients	128	134	6	4,68	95,32
Total vial numbers used	187	202	15	8, 02	91, 98

## Data Availability

The data used in the study were obtained from Private Metro Hospital, which has the largest neonatal intensive care unit in the region. Records of patient information, patient birth weight, and arrival time of the patients were taken. The data used to support the findings of this study are restricted by the Metro Hospital in order to protect patient privacy.
